The article "Minibatch Recursive Least Squares Q-Learning" was published in 2021. Journal: Comput Intell Neurosci.

# Minibatch Recursive Least Squares Q-Learning

**DOI:** 10.1155/2021/5370281

**Published:** 2021-10-08

**Authors:** Chunyuan Zhang, Qi Song, Zeng Meng

**Affiliations:** School of Computer Science and Technology, Hainan University, Haikou, Hainan 570228, China

## Abstract

The deep Q-network (DQN) is one of the most successful reinforcement learning algorithms, but it has some drawbacks such as slow convergence and instability. In contrast, the traditional reinforcement learning algorithms with linear function approximation usually have faster convergence and better stability, although they easily suffer from the curse of dimensionality. In recent years, many improvements to DQN have been made, but they seldom make use of the advantage of traditional algorithms to improve DQN. In this paper, we propose a novel Q-learning algorithm with linear function approximation, called the minibatch recursive least squares Q-learning (MRLS-Q). Different from the traditional Q-learning algorithm with linear function approximation, the learning mechanism and model structure of MRLS-Q are more similar to those of DQNs with only one input layer and one linear output layer. It uses the experience replay and the minibatch training mode and uses the agent's states rather than the agent's state-action pairs as the inputs. As a result, it can be used alone for low-dimensional problems and can be seamlessly integrated into DQN as the last layer for high-dimensional problems as well. In addition, MRLS-Q uses our proposed average RLS optimization technique, so that it can achieve better convergence performance whether it is used alone or integrated with DQN. At the end of this paper, we demonstrate the effectiveness of MRLS-Q on the CartPole problem and four Atari games and investigate the influences of its hyperparameters experimentally.

## 1. Introduction

Reinforcement learning (RL) is an important machine learning methodology for solving sequential decision-making problems. In theory, by interacting with an initially unknown environment, the RL agent can learn the optimal action policies at different states to maximize the cumulative expected return [1]. Unfortunately, in the past several decades, due to the so-called “curse of dimensionality,” RL can only be used to solve some real-world problems with the small-scale discrete or low-dimensional continuous state space. It is not until 2013 that this dilemma was partially solved by Mnih et al. [2]. By combining the Q-learning algorithm with deep learning, they proposed the preliminary version of the deep Q-network (DQN) algorithm. Two years later, Mnih et al. [3] presented the normal version of DQN, which achieves the human-level performance on 49 classical Atari games. Since then, DQN has attracted more and more research attention, and many other novel deep RL algorithms [4, 5] and new applications [6, 7] have been proposed, and thus deep RL has become a thriving research branch in artificial intelligence. However, although DQN has succeeded in some more complicated problems [8–10], it still has many drawbacks, such as slow convergence, instability, and low sample efficiency. Therefore, we will focus on how to improve the DQN's performance in this paper.

The article "Minibatch Recursive Least Squares Q-Learning" was published in 2021. Journal: Comput Intell Neurosci.

Currently, there are three main categories of research work on improving DQN. The first category mainly focuses on how to estimate action values accurately. For example, Hasselt et al. [11] proposed the double DQN, which can reduce the observed overestimation by exploiting the idea of double Q-learning. Wang et al. [12] introduced a dueling network architecture, which separately estimates state values and advantage values to improve the policy evaluation. Hausknecht and Stone [13] presented the deep recurrent Q-network, which is more suitable for solving partial observation problems, by adding recurrent LSTM layers to convolutional networks. Kim et al. [14] combined the mellowmax method with DQN to calculate the target action values, preventing overestimation effectively. Anschel et al. [15] proposed the averaged DQN, which uses some previously learned action-value estimates to produce the current action value. This algorithm can reduce the approximation error variance in the target values. The second category mainly focuses on how to explore or exploit samples efficiently. Schaul et al. [16] presented a prioritized experience replay, which can make the effective use of historical samples to improve the DQN's convergence performance. Fortunato et al. [17] proposed the noisynet DQN, which adds noise to the deep network parameters for aiding efficient exploration. Lee et al. [18] introduced an episodic backward update to improve the sample efficiency. The third category mainly focuses on how to reduce memory and computation. Mnih et al. [19] proposed asynchronous variants of four standard reinforcement learning algorithms, such as the asynchronous one-step Q-learning algorithm and the asynchronous n-step Q-learning algorithm. Interestingly, this work also opens the door to research the asynchronous advantage actor-critic (A3C) algorithm.

In traditional RL, Q-learning algorithms often use linear functions to approximate action values, which have better stability and fewer hyperparameters to be trained than DQNs [20]. In particular, the least squares (LS) type RL algorithms, such as the least squares policy iteration (LSPI) algorithm [21], the fitted-Q iteration (FQI) algorithm [22], and the recursive least squares temporal difference with forgetting factor (RLS-TD-f) algorithm [23], not only have better stability but also have faster convergence. In the research community of adaptive filtering, the LS and the recursive least squares (RLS) algorithms are famous for their fast convergence rate. Obviously, the success of LS-type RL algorithms mainly benefits from this merit. In recent years, many new machine learning algorithms, such as the extreme learning machine (ELM) [24] and the broad learning system [25, 26], have been proposed by combining LS or RLS algorithms. In practice, the last layer of the neural network used for DQN is usually a linear layer, which means that we probably can improve the DQN's performance by integrating DQN with the LS-type RL algorithms. In fact, Levine et al. [20] proposed a hybrid approach—the least squares deep Q-network (LS-DQN), which combines DQN with LSPI or FQI. By retraining the last layer of the policy network with a batch least squares update periodically, LS-DQN can obtain better convergence performance than DQN, whereas LS-DQN is not easy to use. At each update by using LSPI or FQI, LS-DQN needs to use the current network parameters to generate a training dataset, which requires running a forward pass of the deep network for each sample in the experience replay buffer. In addition, LS-DQN needs to generate new state-action features and compute the matrix inverse. From the DQN's learning mechanism, a perfect integrated LS-type algorithm should be able to use the inputs of the DQN's last layer for approximating action values and should have the same learning mode as DQN.

The article "Minibatch Recursive Least Squares Q-Learning" was published in 2021. Journal: Comput Intell Neurosci.

In our previous work [27], we propose two policy control algorithms called ESNRLS-Q and ESNRLS-Sarsa. They seem to meet the above requirements to some extent, although they are also difficult to integrate with DQNs. They use the same experience replay and minibatch learning mode as DQN. In addition, they can avoid computing the matrix inverse and are more suitable for online learning by using recursive least squares (RLS). Based on this work and inspired by the work of Levine et al., we propose a novel minibatch RLS Q-learning algorithm with linear function approximation, called the MRLS-Q. Our main contributions are as follows. (1) By borrowing the experience replay to remove the temporal correlation between the observed transitions, we first combine the traditional Q-learning algorithm with the RLS optimization technique. (2) By using state features rather than state-action features for linear function approximation, we make MRLS-Q able to be used alone and also be integrated into DQN seamlessly. (3) In order to reduce the computational complexity and make the RLS method suitable for training parameters in the minibatch mode, we present an average approximation method for updating the RLS autocorrelation matrix. (4) In order to alleviate the feature change of the same state and integrate MRLS-Q into DQN, we present a new method to define the feature function of MRLS-Q. (5) We demonstrate the effectiveness of MRLS-Q, alone and as the last layer of DQN, by using the CartPole problem and four Atari games, respectively. We also test the influences of its hyperparameters experimentally.

The article "Minibatch Recursive Least Squares Q-Learning" was published in 2021. Journal: Comput Intell Neurosci.

The remainder of this paper is organized as follows.  Section 2 describes the related theories and algorithms of MRLS-Q.  Section 3 represents the detailed derivation and the practical implementation of MRLS-Q. Then, in Section 4, comparison experiments on the CartPole problem and four Atari games are conducted to separately verify the effectiveness of MRLS-Q used alone and as the last layer of DQN. Finally, Section 5 summarizes the whole paper.

## 2. Background

In this section, we briefly review the related theories and algorithms of our MRLS-Q, including the Markov decision process (MDP), DQN, and LS-DQN. In addition, we also describe some notations that will be used throughout this paper.

### 2.1. Markov Decision Process

In RL, a sequential decision problem is generally formulated as an MDP with a five-tuple 〈*𝒮*, *𝒜*, *P*, *r*, *γ*〉, where *𝒮* is the state space, *𝒜* is the action space, *P*(**s**_*t*_′*| ***s**_*t*_, *a*_*t*_) ∈ [0,1] and *r*(**s**_*t*_′*| ***s**_*t*_, *a*_*t*_) ∈ ℛ are the state-transition probability and the immediate reward from the state **s**_*t*_ to the next state **s**_*t*_′ by taking the action *a*_*t*_, and *γ* ∈ (0,1] is the discount factor. At the state **s**_*t*_, the agent's action *a*_*t*_ is determined by the control policy *π*.

For a given MDP, the goal of RL is to learn the optimal policy *π*^*∗*^ for maximizing the cumulative expected return *J*(*π*), i.e.,

(1) $$\begin{array}{c} \pi^{*}=\underset{\pi }{\arg\max}J\left(\pi \right), \end{array}$$

where *J*(*π*) is usually defined in the form of discount return [1] as

(2) $$\begin{array}{c} J\left(\pi \right)=E\left[\sum_{t=0}^{\infty }\gamma^{t}r_{t}|s_{0},\pi \right], \end{array}$$

where **s**_0_ is the initial state, whereas *J*(*π*) is hardly calculated by using the above equation directly, since *P*(**s**_*t*_′*| ***s**_*t*_, *a*_*t*_) is unknown in RL, and **s**_*t*_′ and *r*_*t*_ can only be obtained by the agent's interaction with the environment.

To tackle this problem, RL usually resorts to estimating the action value *Q*^*π*^(**s**_*t*_, *a*_*t*_) to measure the performance of *π* when the initial state and action are **s**_*t*_ and *a*_*t*_. In this paper, we assume that *𝒮* is continuous and *𝒜* is discrete. For this kind of MDP problems, to overcome the curse of dimensionality, *Q*^*π*^(**s**_*t*_, *a*_*t*_) is often approximated by linear function approximators or deep neural networks.

The article "Minibatch Recursive Least Squares Q-Learning" was published in 2021. Journal: Comput Intell Neurosci.

### 2.2. The DQN Algorithm

DQN is probably the most important algorithm in deep RL. It combines the Q-Learning algorithm with deep neural networks and uses the experience relay for breaking the correlation among samples and training network parameters.

The DQN algorithm can be summarized as follows. At the current step *t*, the agent firstly uses the *ϵ*-greedy policy to select the action *a*_*t*_ as

(3) $$\begin{array}{c} a_{t}=\left\{\begin{array}{cc} \underset{a\in A}{\arg\max}Q\left(s_{t},a;\Theta_{t-1}\right), & \text{w.p. }1-\epsilon ,\\ \text{a random action in }A, & \text{w.p. }\epsilon , \end{array}\right. \end{array}$$

where *ϵ* is the exploration factor, Θ_*t*−1_ is the policy network parameter, and *Q*(**s**_*t*_, *a*; Θ_*t*−1_) is approximated by this network. Then, after taking *a*_*t*_, the agent moves to the next state **s**_*t*_′, obtains the reward *r*_*t*_, and stores (**s**_*t*_, *a*_*t*_, **s**_*t*_′, *r*_*t*_, *d*_*t*_) into the experience replay buffer *𝒟*, where *d*_*t*_ ∈ {0,1} denotes that **s**_*t*_′ is the terminal state or not. Next, by using the minibatch $ℳ{\;}_{t}={\left\{\left({\hat{s}}_{t,i},{\hat{a}}_{t,i},{\hat{s}}_{t,i}^{\prime },{\hat{r}}_{t,i},{\hat{d}}_{t,i}\right)\right\}}_{i=1,\ldots ,M}$ sampled from *𝒟* randomly, the algorithm calculates the loss of the policy network as

(4) $$\begin{array}{c} L\left(\Theta_{t-1}\right)=\frac{1}{2M}{\left\|Q^{\pi }\left({\hat{S}}_{t},{\hat{a}}_{t}\right)-Q\left({\hat{S}}_{t},{\hat{a}}_{t};\Theta_{t-1}\right)\right\|}_{2}^{2}, \end{array}$$

where ${\hat{S}}_{t}={\left[{\hat{s}}_{t,1},\ldots ,{\hat{s}}_{t,M}\right]}^{T}$, ${\hat{a}}_{t}={\left[{\hat{a}}_{t,1},\ldots ,{\hat{a}}_{t,M}\right]}^{T}$, and $Q^{\pi }\left({\hat{S}}_{t},{\hat{a}}_{t}\right)$ is the target value of $Q\left({\hat{S}}_{t},{\hat{a}}_{t};\Theta_{t-1}\right)$, which is estimated by the target network as

(5) $$\begin{array}{c} Q^{\pi }\left({\hat{S}}_{t},{\hat{a}}_{t}\right)={\hat{r}}_{t}+\gamma \left(1-{\hat{d}}_{t}\right)\circ \underset{a\in A}{\max}Q\left({\hat{S}}_{t}^{\prime },a;\tilde{\Theta }\right), \end{array}$$

where ${\hat{r}}_{t}={\left[{\hat{r}}_{t,1},\ldots ,{\hat{r}}_{t,M}\right]}^{T}$, ${\hat{S}}_{t}^{\prime }={\left[{\hat{s}}_{t,1}^{\prime },\ldots ,{\hat{s}}_{t,M}^{\prime }\right]}^{T}$, ${\hat{d}}_{t}={\left[{\hat{d}}_{t,1},\ldots ,{\hat{d}}_{t,M}\right]}^{T}$, ∘ denotes the Hadamard product, and $\tilde{\Theta }$ is the target network parameter which is copied from the policy network every some fixed steps or episodes. Finally, by using some gradient descent optimization method, the algorithm updates Θ_*t*−1_ to Θ_*t*_. For example, by using the SGD method [28], Θ_*t*−1_ is updated as

(6) $$\begin{array}{c} \Theta_{t}=\Theta_{t-1}-\alpha \nabla_{\Theta_{t-1}}, \end{array}$$

where *α* is the learning rate and ∇_Θ_*t*−1__ denotes ∂*L*(Θ_*t*−1_)/∂Θ_*t*−1_.

The article "Minibatch Recursive Least Squares Q-Learning" was published in 2021. Journal: Comput Intell Neurosci.

### 2.3. The LS-DQN Algorithm

LS-DQN is a hybrid approach, which combines the traditional LSPI or FQI algorithm with the DQN algorithm. By enjoying the stability and efficiency of LSPI or FQI, it can obtain better performance than DQN.

The LS-DQN algorithm can be briefly summarized as follows. Whenever the agent runs DQN some steps, it uses LSPI or FQI to retrain the last layer of the policy network once. The retraining consists of the following three substeps. Firstly, by recalculating all samples in the experience replay buffer with the current network parameters, the policy network generates a new dataset $\tilde{𝒟}$. Secondly, by using the current network parameters and the dataset $\tilde{𝒟}$, the algorithm generates state-action features. Finally, the algorithm uses LSPI to retrain the current last-layer parameter Θ_*t*_^*L*^ in the policy network as

(7) $$\begin{array}{c} {\left[{\left(\Theta_{t\left(:,1\right)}^{L}\right)}^{T},\ldots ,{\left(\Theta_{t\left(:,\left|A\right|\right)}^{L}\right)}^{T}\right]}^{T}=A^{-1}b, \end{array}$$

where Θ_*t*(:,*i*)_^*L*^ is the *i*^th^ column vector of Θ_*t*_^*L*^. Besides, *A* and **b** are defined as follows:

(8) $$\begin{array}{c} A=\frac{1}{\left|\tilde{D}\right|}\sum_{j=1}^{\left|\tilde{D}\right|}\left[\phi \left({\hat{s}}_{j},{\hat{a}}_{j}\right){\left(\phi \left({\hat{s}}_{j},{\hat{a}}_{j}\right)-\gamma \left(1-d_{j}\right)\phi \left({\hat{s}}_{j}^{\prime },\pi \left({\hat{s}}_{j}^{\prime }\right)\right)\right)}^{T}\right],\\ b=\frac{1}{\left|\tilde{D}\right|}\sum_{j=1}^{\left|\tilde{D}\right|}\left[\phi \left({\hat{s}}_{j},{\hat{a}}_{j}\right)r_{j}\right], \end{array}$$

where $\phi \left({\hat{s}}_{j},{\hat{a}}_{j}\right)$ is the state-action feature of the state-action pair $\left({\hat{s}}_{j},{\hat{a}}_{j}\right)$. As Levine et al. stated in their work [20], the algorithm can also retrain Θ_*t*_^*L*^ by using FQI, since it is a batch shallow RL algorithm that computes iterative approximations of the Q-function using regression. For brevity, we will not discuss the FQI algorithm in this paper.

## 3. The Proposed Algorithm

In this section, we will introduce the detailed derivation and the practical implementation of our proposed algorithm, respectively. Our algorithm, the MRLS-Q algorithm, can be used not only alone but also as the last layer of DQN.

The article "Minibatch Recursive Least Squares Q-Learning" was published in 2021. Journal: Comput Intell Neurosci.

### 3.1. Algorithm Derivation

MRLS-Q is a new Q-learning algorithm with linear function approximation, but it is more similar to the DQN algorithm rather than the traditional Q-learning algorithm. It uses the experience replay and the minibatch training mode, separates the linear function approximator into a policy approximator and a target approximator, and uses the state features rather than the state-action features. Besides, it uses an average RLS method for updating parameters.

First, we introduce the agent's interaction with the environment. At the current step *t*, the agent also uses the *ϵ*-greedy policy to select the action *a*_*t*_ as equation (3). Note here that *Q*(**s**_*t*_, *a*; Θ_*t*−1_) is approximated by the policy approximator as

(9) $$\begin{array}{c} Q\left(s_{t},a;\Theta_{t-1}\right)=\phi {\left(s_{t}\right)}^{T}\Theta_{t-1\left(:,\text{in}\left(a\right)\right)}, \end{array}$$

where *ϕ*(**s**_*t*_) ∈ ℛ^*N*^ is the feature vector of **s**_*t*_, Θ_*t*−1_ ∈ ℛ^*N* × |*𝒜*|^ is the policy approximator parameter, in(*a*) denotes the index of *a* in *𝒜*, and Θ_*t*−1(:,in(*a*))_ is the in(*a*)^th^ column vector of Θ_*t*−1_. Then, the agent takes *a*_*t*_, moves to **s**_*t*_′, obtains *r*_*t*_, and stores (**s**_*t*_, *a*_*t*_, **s**_*t*_′, *r*_*t*_, *d*_*t*_) into the experience replay buffer *𝒟*.

Second, we introduce the RLS update of the policy approximator parameter in the minibatch training mode. Let $ℳ{\;}_{n}={\left\{\left({\hat{s}}_{n,i},{\hat{a}}_{n,i},{\hat{s}}_{n,i}^{\prime },{\hat{r}}_{n,i},{\hat{d}}_{n,i}\right)\right\}}_{i=1,\ldots ,M}$ denote the minibatch sampled from *𝒟* at the *n*^th^ step, and let $\Phi \left({\hat{S}}_{n}\right)={\left[\phi \left({\hat{s}}_{n,1}\right),\ldots ,\phi \left({\hat{s}}_{n,M}\right)\right]}^{T}$ denote the feature matrix of ${\hat{S}}_{n}$. Define the least squares loss function as

(10) $$\begin{array}{c} \hat{L}\left(\Theta \right)=\frac{1}{2M}\sum_{n=1}^{t}\lambda^{t-n}{\left\|Q^{\pi }\left({\hat{S}}_{n},{\hat{a}}_{n}\right)-Q\left({\hat{S}}_{n},{\hat{a}}_{n};\Theta \right)\right\|}_{2}^{2}, \end{array}$$

where *λ* ∈ (0,1] is the forgetting factor and $Q\left({\hat{S}}_{n},{\hat{a}}_{n};\Theta \right)$ is approximated by the policy approximator as

(11) $$\begin{array}{c} Q\left({\hat{S}}_{n},{\hat{a}}_{n};\Theta \right)=\Phi \left({\hat{S}}_{n}\right)\Theta_{\left(:,\text{in}\left({\hat{a}}_{n}\right)\right)}, \end{array}$$

and $Q^{\pi }\left({\hat{S}}_{n},{\hat{a}}_{n}\right)$ is estimated by the target approximator as

(12) $$\begin{array}{c} Q^{\pi }\left({\hat{S}}_{n},{\hat{a}}_{n}\right)={\hat{r}}_{n}+\gamma \left.\left(1-{\hat{d}}_{n}\right)\right)\circ \underset{a\in A}{\max}\Phi \left({\hat{S}}_{n}^{\prime }\right){\tilde{\Theta }}_{\left(:,\text{in}\left(a\right)\right)}, \end{array}$$

where $\tilde{\Theta }$ is the target approximator parameter which is copied from the policy approximator every some fixed steps or episodes. Then, the parameter learning problem of the policy approximator can be transformed into

(13) $$\begin{array}{c} \Theta_{t}=\underset{\Theta }{\arg\min}\hat{L}\left(\Theta \right). \end{array}$$

By using the chain rule, we can get

(14) $$\begin{array}{c} {\hat{\nabla }}_{\Theta }=-\frac{1}{M}\sum_{n=1}^{t}\lambda^{t-n}{\left(\Phi \left({\hat{S}}_{n}\right)\right)}^{T}\left({\hat{Q}}^{\pi }\left({\hat{S}}_{n},A\right)-\hat{Q}\left({\hat{S}}_{n},A;\Theta \right)\right), \end{array}$$

where ${\hat{\nabla }}_{\Theta }$ denotes $\partial \hat{L}\left(\Theta \right)/\partial \Theta$, and an element in $\hat{Q}\left({\hat{S}}_{n},𝒜;\Theta \right)\in {ℛ}^{M\times \left|𝒜\right|}$ is defined as

(15) $$\begin{array}{c} \hat{Q}\left({\hat{s}}_{n,i},a;\Theta \right)=\left\{\begin{array}{cc} Q\left({\hat{s}}_{n,i},{\hat{a}}_{n,i};\Theta \right), & a={\hat{a}}_{n,i},\\ 0, & a\neq {\hat{a}}_{n,i}, \end{array}\right. \end{array}$$

and an element in ${\hat{Q}}^{\pi }\left({\hat{S}}_{n},𝒜\right)\in {ℛ}^{M\times \left|𝒜\right|}$ is defined as

(16) $$\begin{array}{c} {\hat{Q}}^{\pi }\left({\hat{s}}_{n,i},a\right)=\left\{\begin{array}{cc} Q^{\pi }\left({\hat{s}}_{n,i},{\hat{a}}_{n,i}\right), & a={\hat{a}}_{n,i},\\ 0, & a\neq {\hat{a}}_{n,i}. \end{array}\right. \end{array}$$

Let ${\hat{\nabla }}_{\Theta }=0$. Then, we can get

(17) $$\begin{array}{c} \Theta_{t}=A_{t}^{-1}B_{t}, \end{array}$$

where

(18) $$\begin{array}{c} A_{t}=\frac{1}{M}\sum_{n=1}^{t}\lambda^{t-n}{\left(\Phi \left({\hat{S}}_{n}\right)\right)}^{T}\Phi \left({\hat{S}}_{n}\right),\\ B_{t}=\frac{1}{M}\sum_{n=1}^{t}\lambda^{t-n}{\left(\Phi \left({\hat{S}}_{n}\right)\right)}^{T}{\hat{Q}}^{\pi }\left({\hat{S}}_{n},A\right). \end{array}$$

Rewrite the above two equations as the following recursive forms:

(19) $$\begin{array}{c} A_{t}=\lambda A_{t-1}+\frac{1}{M}{\left(\Phi \left({\hat{S}}_{t}\right)\right)}^{T}\Phi \left({\hat{S}}_{t}\right), \end{array}$$

(20) $$\begin{array}{c} B_{t}=\lambda B_{t-1}+\frac{1}{M}{\left(\Phi \left({\hat{S}}_{t}\right)\right)}^{T}{\hat{Q}}^{\pi }\left({\hat{S}}_{t},A\right). \end{array}$$

Further, rewrite the above two equations as the following vector forms:

(21) $$\begin{array}{c} A_{t}=\lambda A_{t-1}+\frac{1}{M}\sum_{i=1}^{M}\phi \left({\hat{s}}_{t,i}\right){\left(\phi \left({\hat{s}}_{t,i}\right)\right)}^{T}, \end{array}$$

(22) $$\begin{array}{c} B_{t}=\lambda B_{t-1}+\frac{1}{M}\sum_{i=1}^{M}\phi \left({\hat{s}}_{t,i}\right){\hat{Q}}^{\pi }\left({\hat{s}}_{t,i},A\right), \end{array}$$

where ${\hat{Q}}^{\pi }\left({\hat{s}}_{t,i},𝒜\right)$ is the *i*^th^ row vector of ${\hat{Q}}^{\pi }\left({\hat{S}}_{t},𝒜\right)$. Unfortunately, we cannot directly use the Sherman–Morrison formula [29] to compute *A*_*t*_^−1^, since the last term in the right-hand side of equation (21) is a sum of vector products.

The article "Minibatch Recursive Least Squares Q-Learning" was published in 2021. Journal: Comput Intell Neurosci.

Next, we present an average approximation method to deal with the above problem. Considering that all training samples are from the same environment and thus their features have some similarity, we rewrite equations (21) and (22) as follows:

(23) $$\begin{array}{c} A_{t}\approx \lambda A_{t-1}+k{\bar{\phi }}_{t}{\bar{\phi_{t}}}^{T}, \end{array}$$

(24) $$\begin{array}{c} B_{t}\approx \lambda B_{t-1}+k{\bar{\phi }}_{t}{\bar{q}}_{t}^{\pi }, \end{array}$$

where *k* is the approximation factor, and ${\bar{\phi }}_{t}$ and ${\bar{q}}_{t}^{\pi }$ are defined as

(25) $$\begin{array}{c} {\bar{\phi }}_{t}=\frac{1}{M}\sum_{i=1}^{M}\phi \left({\hat{s}}_{t,i}\right), \end{array}$$

(26) $$\begin{array}{c} {\bar{q}}_{t}^{\pi }=\frac{1}{M}\sum_{i=1}^{M}{\hat{Q}}^{\pi }\left({\hat{s}}_{t,i},A\right). \end{array}$$

Let *P*_*t*_=*A*_*t*_^−1^. By using the Sherman–Morrison formula for (23), we can get

(27) $$\begin{array}{c} P_{t}=\frac{1}{\lambda }\left(P_{t-1}-g_{t}v_{t}^{T}\right), \end{array}$$

where

(28) $$\begin{array}{c} v_{t}=P_{t-1}{\bar{\phi }}_{t}, \end{array}$$

(29) $$\begin{array}{c} g_{t}=\frac{kv_{t}}{\lambda +kv_{t}^{T}{\bar{\phi }}_{t}}. \end{array}$$

Plugging equations (24) and (27) into (17), we finally get

(30) $$\begin{array}{c} \Theta_{t}\approx \Theta_{t-1}+\frac{kP_{t-1}{\bar{\phi }}_{t}\left({\bar{q}}_{t}^{\pi }-{\bar{q}}_{t}\right)}{\lambda +kv_{t}^{T}{\bar{\phi }}_{t}}, \end{array}$$

where

(31) $$\begin{array}{c} {\bar{q}}_{t}=\frac{1}{M}\sum_{i=1}^{M}\hat{Q}\left({\hat{s}}_{t,i},A;\Theta_{t-1}\right), \end{array}$$

where $\hat{Q}\left({\hat{s}}_{t,i},𝒜;\Theta_{t-1}\right)$ denotes the *i*^th^ row vector of $\hat{Q}\left({\hat{S}}_{t},𝒜;\Theta_{t-1}\right)$.

### 3.2. Practical Implementation

As reviewed in Section 2.2, DQN generally uses gradient descent methods to update network parameters. To make MRLS-Q easier to be integrated into DQN, we next rewrite equation (30) as the “gradient descent” form of ∇_Θ_*t*−1__.

If the loss function of MRLS-Q is defined by equation (4), by using the chain rule for equation (4), we can get

(32) $$\begin{array}{c} \nabla_{\Theta_{t-1}}=-\frac{1}{M}{\left(\Phi \left({\hat{S}}_{t}\right)\right)}^{T}\left({\hat{Q}}^{\pi }\left({\hat{S}}_{t},A\right)-\hat{Q}\left({\hat{S}}_{t},A;\Theta_{t-1}\right)\right). \end{array}$$

Recall the fact that we once used $k{\bar{\phi }}_{t}{\bar{\phi_{t}}}^{T}$ and $k{\bar{\phi }}_{t}{\bar{q}}_{t}^{\pi }$ in equations (23) and (24) to replace $\left(1/M\right){\left(\Phi \left({\hat{S}}_{t}\right)\right)}^{T}\Phi \left({\hat{S}}_{t}\right)$ and $\left(1/M\right){\left(\Phi \left({\hat{S}}_{t}\right)\right)}^{T}{\hat{Q}}^{\pi }\left({\hat{S}}_{t},𝒜\right)$ in equations (19) and (20), respectively, which means

(33) $$\begin{array}{c} k{\bar{\phi }}_{t}{\bar{\phi_{t}}}^{T}=\frac{1}{M}{\left(\Phi \left({\hat{S}}_{t}\right)\right)}^{T}\Phi \left({\hat{S}}_{t}\right), \end{array}$$

(34) $$\begin{array}{c} k{\bar{\phi }}_{t}{\bar{q}}_{t}^{\pi }=\frac{1}{M}{\left(\Phi \left({\hat{S}}_{t}\right)\right)}^{T}{\hat{Q}}^{\pi }\left({\hat{S}}_{t},A\right). \end{array}$$

In addition, from equation (31), we can obtain

(35) $$\begin{array}{c} k{\bar{\phi }}_{t}{\bar{q}}_{t}=\frac{k}{M}{\bar{\phi }}_{t}\sum_{i=1}^{M}\hat{Q}\left({\hat{s}}_{t,i},A;\Theta_{t-1}\right). \end{array}$$

Using equation (9) yields

(36) $$\begin{array}{c} \hat{Q}\left({\hat{s}}_{t,i},A;\Theta_{t-1}\right)=\phi {\left({\hat{s}}_{t,i}\right)}^{T}\Theta_{t-1}. \end{array}$$

Then, equation (35) can be written as

(37) $$\begin{array}{c} k{\bar{\phi }}_{t}{\bar{q}}_{t}=\frac{k}{M}{\bar{\phi }}_{t}\sum_{i=1}^{M}\phi {\left({\hat{s}}_{t,i}\right)}^{T}\Theta_{t-1}. \end{array}$$

Further, from equation (25), the above equation can be written as

(38) $$\begin{array}{c} k{\bar{\phi }}_{t}{\bar{q}}_{t}=k{\bar{\phi }}_{t}{\bar{\phi }}_{t}^{T}\Theta_{t-1}. \end{array}$$

Next, plugging equation (33) into equation (38), we have

(39) $$\begin{array}{c} k{\bar{\phi }}_{t}{\bar{q}}_{t}=\frac{1}{M}{\left(\Phi \left({\hat{S}}_{t}\right)\right)}^{T}\Phi \left({\hat{S}}_{t}\right)\Theta_{t-1}. \end{array}$$

From equations (9) and (11), the above equation can be rewritten as

(40) $$\begin{array}{c} k{\bar{\phi }}_{t}{\bar{q}}_{t}=\frac{1}{M}{\left(\Phi \left({\hat{S}}_{t}\right)\right)}^{T}Q\left({\hat{s}}_{t,i},A;\Theta_{t-1}\right). \end{array}$$

Using equations (34) and (40), we can get

(41) $$\begin{array}{c} k{\bar{\phi }}_{t}\left({\bar{q}}_{t}^{\pi }-{\bar{q}}_{t}\right)=-\nabla_{\Theta_{t-1}}. \end{array}$$

Therefore, we can rewrite equation (30) as

(42) $$\begin{array}{c} \Theta_{t}\approx \Theta_{t-1}-\frac{P_{t-1}}{\lambda +kv_{t}^{T}{\bar{\phi }}_{t}}\nabla_{\Theta_{t-1}}. \end{array}$$

It shows that $\left(P_{t-1}/\left(\lambda +kv_{t}^{T}{\bar{\phi }}_{t}\right)\right)$ is the learning rate of Θ_*t*_ in MRLS-Q.

The article "Minibatch Recursive Least Squares Q-Learning" was published in 2021. Journal: Comput Intell Neurosci.

However, although RLS has a fast convergence rate, it often suffers from overfitting. In recent years, there has been extensive research on this problem. Based on Ekşioğlu's work [30], we add an *L*_1_ regularization term into the above equation, i.e.,

(43) $$\begin{array}{c} \Theta_{t}\approx \Theta_{t-1}-\frac{P_{t-1}}{\lambda +kv_{t}^{T}{\bar{\phi }}_{t}}\nabla_{\Theta_{t-1}}-\eta P_{t}\mathrm{sgn}\left(\Theta_{t-1}\right), \end{array}$$

where *η* is the regularization factor and sgn(·) is the sign function.

Based on the above derivation, the pseudocode of MRLS-Q is summarized in Algorithm 1, and the flow diagram of MRLS-Q is summarized in Figure 1. In the practical implementation, here ∇_Θ_*t*−1__ can be calculated by the automatic differentiation package of PyTorch or TensorFlow directly. Besides being used alone, MRLS-Q can also be used as the last layer of DQN, since it uses the same loss function and experience replay as DQN. However, there is still an obstacle to the combination of MRLS-Q and DQN. As the training goes on, the parameters of the DQN network are continuously changing, and the outputs of the same inputs are changing as well. Thus, we cannot use the inputs of the DQN's last layer as the features of MRLS-Q directly. In order to alleviate this kind of change and integrate MRLS-Q into DQN, we present a new method to define the feature function of MRLS-Q as

(44) $$\begin{array}{c} \Phi \left({\hat{S}}_{n}\right)=\frac{X_{t}^{L}}{\left(1/MN_{L-1}\right)\sum_{i=1}^{M}\sum_{j=1}^{N_{L-1}}X_{t,i,j}^{L}+\nu }, \end{array}$$

where *X*_*t*_^*L*^ ∈ ℛ^*M*×*N*_*L*−1_^ is the output matrix of the DQN's penultimate layer and *ν* is a small hyperparameter to prevent the denominator becoming zero.

## 4. Experiments

In this section, we use two sets of experiments to demonstrate the effectiveness of MRLS-Q. Our experiments are divided into two sections. In Section 4.1, we test MRLS-Q on the CartPole problem as an independent algorithm. In Section 4.2, we test MRLS-Q on four Atari games as the last layer of DQN.

### 4.1. The CartPole Problem

In this set of experiments, we firstly verify the performance of MRLS-Q on the CartPole-v0 problem, which is from the OpenAI Gym. For comparison purposes, we build a new algorithm called Adam-Q, by replacing $P_{t-1}/\left(\lambda +kv_{t}^{T}{\bar{\phi }}_{t}\right)$ in equation (42) with the Adam optimizer, since the traditional Q-learning algorithm with linear function approximation is hardly convergent in 100 episodes. Then, we verify the influences of hyperparameters on MRLS-Q, experimentally.

To compare the performance between MRLS-Q and Adam-Q, the experimental settings are summarized as follows. (1) Both algorithms use 400 radial basis functions (RBFs) for action-value approximation. These RBFs are generated from 10^4^ random samples in the CartPole's state space, by using eight scikit-learn RBFSamplers [31] with kernel parameters {0.5, 1.0, 1.5, 2.0, 2.5, 3.0, 3.5, 4.0}. (2) The exploration rate *ϵ* is initialized to 0.95 and is gradually decreased to 0.01 over 1000 steps. (3) The discount factor *γ* is 0.99. (4) The capacity of the experience replay buffer *𝒟* is 10^4^, and the minibatch size is 32. The learning starts when the number in *𝒟* reaches the minibatch size. (5) The policy approximator parameter Θ_0_ and the target approximator parameter $\tilde{\Theta }$ are initialized randomly. (6) $\tilde{\Theta }$ is updated by Θ_*t*_ each step. Note that the performances of both algorithms will get worse if we increase the update steps, since the CartPole problem is very simple and both algorithms converge fast. (7) The max norm of ∇_Θ_*t*−1__ is clipped to 1 by the *L*_2_ norm. (8) The two algorithms run five times and 100 episodes for each time. In each episode, each algorithm runs 200 steps at most. (9) Besides, in Adam-Q, the learning rate, *β*_1_, and *β*_2_ of Adam are 0.001, 0.9, and 0.999; in MRLS-Q, the initialization *P*_0_, the forgetting factor *λ*, the regularization factor *η*, and the approximation factor *k* are 0.5*I*, 1, 10^−5^, and 1/32, respectively. The average result of this experiment is shown in Figure 2(a). It can be seen that our MRLS-Q has better convergence than Adam-Q.

The article "Minibatch Recursive Least Squares Q-Learning" was published in 2021. Journal: Comput Intell Neurosci.

To investigate hyperparameter influences on MRLS-Q, we test |*𝒟*| ∈ {500,1000,5000,10000}, *P*_0_ ∈ {0.1*I*, 0.2*I*, 0.5*I*, *I*}, and *k* ∈ {(1/2), (1/8), (1/32), (1/128)}, respectively. The other settings of these experiments are the same as what we did for MRLS-Q in the previous experiment. The average results of these experiments are presented in Figures 2(b)–2(d). From Figure 2(b), it shows that the capacity of *𝒟* has a significant influence on the performance of MRLS-Q. The larger capacity will result in the better performance, since big *𝒟* is helpful to remove the correlation between the observed transitions. From Figure 2(c), it can be seen that MRLS-Q is robust to the initialization *P*_0_, whereas too big *P*_0_ will make MRLS-Q become unstable and too small *P*_0_ will make MRLS-Q converge slowly. From Figure 2(d), it can be seen that *k* also has a significant influence on MRLS-Q. From equation (29), bigger *k* will make *P*_*t*_ update with higher strength. If state feature values change greatly, *k* should be set to a big value.

### 4.2. Four Atari Games

In this set of experiments, we verify MRLS-Q as the last layer of DQN on four Atari games: Pong-v0, Breakout-v0, SpaceInvaders-v0, and RiverRaid-v0, which are from the OpenAI Gym. Here we choose the traditional DQN algorithm with the Adam optimizer for comparison. For Adam-DQN and in the second to fifth layers of Hybrid-DQN, the learning rate, *β*_1_, and *β*_2_ of Adam are 0.0000625, 0.9, and 0.999; in the last layer of Hybrid-DQN, the initialization *P*_0_, the forgetting factor *λ*, the regularization factor *η*, the approximation factor *k*, and *ν* are 0.1I, 1, 10^−8^, 1/2, and 10^−12^, respectively. Note that here we use a big *k* to update *P*_*t*_ for adapting to the feature change.

The article "Minibatch Recursive Least Squares Q-Learning" was published in 2021. Journal: Comput Intell Neurosci.

The average evaluation results are presented in Figure 3. It shows that Hybrid-DQN can speed up the convergence of all tested games.  Figure 3(a) is much clearer to demonstrate this advantage, since the Pong game is much simpler than other three games. In addition, Figures 3(a), 3(c), and 3(d) show that Hybrid-DQN can improve the convergence quality of Pong, SpaceInvaders, and RiverRaid, and Figure 3(b) shows that Hybrid-DQN can improve the learning stability of Breakout. In summary, by integrating our MRLS-Q, Hybrid-DQN can improve the stability and performance. Compared with the LS-DQN algorithm, MRLS-Q can be used as the last layer of DQN directly, and thus Hybrid-DQN is easier to use.

## 5. Conclusion

How to improve convergence and stability of the DQN algorithm is one of the key issues in deep RL. In this paper, we propose MRLS-Q, a linear RLS function approximation algorithm with the similar learning mechanism to DQN. MRLS-Q can be used not only alone but also as the last layer of DQN. Similar to LS-DQN, the Hybrid-DQN with MRLS-Q can enjoy rich representations from deep RL networks as well as stability and data efficiency of the RLS method, but it can seamlessly integrate MRLS-Q and thus is easier to use. In MRLS-Q, we use the experience replay to break the correlation between training samples, present an average RLS optimization method to improve the convergence performance and reduce the computational complexity, employ an *L*_1_ regularization technique to prevent overfitting, and propose a new method to define the feature function for alleviating the feature change of the same state and integrating MRLS-Q into DQN. Experiment results on the CartPole problem demonstrate that MRLS-Q has better convergence than Adam-Q and reveal the hyperparameter influences on MRLS-Q. In addition, experiment results on four Atari games demonstrate that DQN can improve convergence and stability by integrating with MRLS-Q.

## Figures and Tables

**Figure 1:** Flow diagram of MRLS-Q.

The article "Minibatch Recursive Least Squares Q-Learning" was published in 2021. Journal: Comput Intell Neurosci.

**Figure 2:** Performance comparison and hyperparameter influences on MRLS-Q. (a) Adam-Q vs. MRLS-Q. (b) Influence of *𝒟*'s capacity. (c) Influence of *P*'s initialization. (d) Influence of *k* value.

**Figure 3:** Performance comparison between Adam-DQN and Hybrid-DQN. (a) Pong. (b) Breakout. (c) SpaceInvaders. (d) RiverRaid.

**Algorithm 1:** MRLS-Q.

## Data Availability

The data used to support the findings of this study are available from the corresponding author upon request.
